The article "Investigating the Impact of Bank Housing Credit Risk Control Strategy by Blockchain Technology on the Household Consumption Plan" was retracted in 2023. Reasons: signs of a paper mill; suspected computer-generated content; unreliable results or conclusions; concerns about the data.

# Investigating the Impact of Bank Housing Credit Risk Control Strategy by Blockchain Technology on the Household Consumption Plan

**DOI:** 10.1155/2022/7021384

**Published:** 2022-07-31

**Authors:** Liang Liu, Shuhong Li

**Affiliations:** ^1^School of Management, Hefei University of Technology, Hefei 230009, China; ^2^Huishang Bank, Hefei 230001, China

## Abstract

It is essential to solve the problem of information asymmetry in bank housing credit management, thus reducing bank operating costs and credit risk. Therefore, the present work constructs a bank housing credit blockchain alliance system based on the technical characteristics of blockchain to strengthen bank housing credit risk control. First, according to blockchain's elements and system architecture, the application of blockchain to bank housing credit business is analyzed. On this basis, the bank housing credit risk control strategy is proposed. Finally, the mathematical model is used to investigate residents' household consumption to explore the impact of housing credit on the household consumption plan of residents. The results show that when the educational level of the head of household is illiterate or semi-illiterate, the coefficients of participation credit (PC), nonparticipation credit (NPC), and total samples (TSs) of total household consumption are −0.064, 0.067, and 0.174, respectively; when the educational level of the head of household is primary school or junior middle school, the coefficients of PC, NPC, and TS of total household consumption are -0.026, 0.017, and 0.105, respectively; when the educational level of the head of household is high school or above, the coefficients of PC, NPC, and TS of total household consumption are 0.084, 0.073, and 0.064, respectively. The results indicate that the education level of the head of household plays a crucial role in the family consumption plan. Those with a high educational level will compromise on the best consumption decision after constantly weighing the consumption motivation and consumption thinking after obtaining the credit funds. The content reported here is vitally significant in guiding households to clarify the proportion of credit fund distribution and understand their consumption tendency.

## 1. Introduction

In recent years, commercial banks have widely expanded their housing loan business with the rapid development of China's real estate industry. The housing loan business has been accumulating and has occupied an important proportion of bank loans. In addition, the loan business in China is highly similar to the Western loan business due to the influence of the West [1]. In 2016, housing loans accounted for 45% of all new loans. In February 2017, the proportion of personal housing loans in new loans decreased by 12.49%. Although housing loans still maintained a growth trend, the growth rate gradually decreased. Various financial institutions began to carry out special management on housing credit and continuously strengthen the supervision of the financial industry to reduce loan risks, which effectively reduced the nonperforming loan ratio of banks [2, 3]. Moreover, major banks have begun to rectify some chaos in the financial loan industry since 2017 to avoid the problem of bank fund idling. Now banks are gradually stricter and standardized in the speed and review of housing loans [4]. Although the current social credit risk control is not perfect, many studies have provided references for it.

Wang and Zhao (2022) reported that there is a risk formation mechanism similar to the subprime mortgage crisis in China's housing credit market. The contradiction between supply and demand of public housing is prominent; the access standards for the housing credit market are loose; the banks providing mortgage loans lack reasonable hedging measures; and the long-term interest rate fluctuations and insufficient liquidity of housing property rights have made China's housing credit market risk accumulating. The authors believe that precautions must be taken to prevent housing credit risks in China [5]. Eerola pointed out that, as an important way for the market economy to allocate resources, the housing credit market is a place where capital and funds are highly concentrated. It is closely related to the development of the national economy and is conducive to promoting economic development and optimizing the industrial structure. At the same time, the housing credit market has great risks. Especially in the current situation where the information is seriously asymmetric and the market is not fully developed, housing credit risks will have a great impact on the healthy development of the housing credit market [6]. The authors studied the relationship between credit growth and house price appreciation by analyzing the macroprudential measures of household debt and systemic risk in various countries. They also used household-level data to carry out policy reforms to further understand the implementation effects and operating mechanisms of these measures [6–8].

As mentioned above, many scholars have carried out research on the solution to credit risk problems, mainly through the construction of a credit risk evaluation system or model to identify credit risk and further manage it. These methods lack certain initiative and cannot fundamentally solve the risk problem brought by housing credit. This work utilizes blockchain technology to control the credit risk and takes S Bank as an example to put forward corresponding strategies and suggestions for the housing credit risk control of banks. The innovation of this study is to adopt blockchain technology to study housing credit risk, providing a relatively safe platform for housing credit and an important guarantee for housing credit. This study offers a reference for improving the security of housing credit and contributes to the elimination of the social credit crisis.

## 2. Bank Housing Credit Risk Control

### 2.1. Block Data Structure and Functional Framework of the Blockchain System

#### 2.1.1. Block Data Structure of Blockchain

Figure 1 reveals the data structure of blockchain.

As can be seen from Figure 1 above, the blockchain is composed of a block header and a block body. The block header includes timestamps, random numbers, target hashes, and Merkle roots. The block header is the main component of each blockchain to effectively identify the blockchain. The block body generates the Merkle root through the Merkle tree data structure and counts it into the block header. This value is unique. The blocks are connected in chronological order to form a blockchain. Each blockchain is connected by the address information of the previous block in the block header to form a data chain with comprehensive transaction records [9].

#### 2.1.2. Overall Functional Architecture of the Blockchain System

In the continuous development of digital technology, the data structure of blockchain is also constantly updated. From the earliest distributed accounting system to Ethereum to the current alliance chain, it can be found that blockchain is constantly integrating with digital technology. Although different blockchains have some specific applications, their overall architecture is almost the same [10].  Figure 2 displays the general functional framework of the system.

As shown in Figure 2, a consortium chain refers to a blockchain jointly managed by multiple institutions. Each organization or institution manages one or more nodes, and its data only allow different institutions in the system to read, write, and send. The read and write rights and bookkeeping rights on the consortium chain are limited by the consortium rules. For example, the blockchain consortium and the Hyperledger project supported by the Linux Foundation, which is participated by more than 40 banks, belong to the consortium chain project.

The advantages of applying blockchain in banks' housing credit business are as follows:

1. Improving the authenticity of preloan investigation
2. The consensus-sharing mechanism based on the blockchain can effectively solve credit problems such as information sharing. The R3 blockchain consortium in the blockchain consortium chain model is most suitable for integration with current financial institutions, so banks can adopt this technology. The consensus mechanism in blockchain technology effectively improves the authenticity and transparency of data in the blockchain and has multiple advantages, such as nontampering and traceability, which helps banks obtain real and effective customer information [11–14].
3. Strengthening the prudence of review in loans
4. The preloan investigation based on blockchain technology can improve the validity, authenticity, and transparency of user information data, effectively avoiding the waste of human resources while ensuring the efficiency of loan review. The advantages brought by the feature of blockchain information sharing are more obvious in bank loans. Banks participating in loans do not need to conduct repeated surveys. In addition, each participating node in the blockchain will add the user's data information and stamp it with time, increasing the plasticity of the data chain [15].
5. Optimizing the effectiveness of postloan management
6. First, the bank can understand the dynamic situation of customers and the flow of funds and other information data based on the blockchain, so it can easily understand the direction of the user's loan. The data determine whether the customer has the economic conditions to repay the principal and interest [16]. Finally, the traceability of blockchain data effectively prevents the bank from repeatedly mortgaged or sold the collateral that has been mortgaged and provides a strong guarantee for the bank's rights and interests [17].

### 2.2. Bank Housing Credit Risk Control Strategy

Figure 3 illustrates the bank's housing credit risk control strategy proposed here.

#### 2.2.1. External Supervision and Internal Control Strategy

External supervision is mainly divided into government financial institutions' custody of banks and the maintenance of real estate trading institutions on developers. The housing credit risk of S Bank often occurs, which may be caused by the low comprehensive quality of banking personnel and inadequate supervision. Given this phenomenon, government financial institutions should establish a housing credit risk control system as soon as possible. Inspired by the mature risk control strategies of foreign markets, the present work selects a comprehensive supervision model with real estate transactions as the platform and government financial regulators as the center. In addition, the housing credit market's operation status and existing risks must be comprehensively tested using the network, information, and human resources. Furthermore, it is necessary to assess the market risk of housing credit objectively and warn of possible dangers timely [18, 19]. Real estate trading institutions should refine the loss-proof system and civil compensation legal procedures to enhance the protection system's operability. In addition, the group litigation system of housing credit dispute cases can be introduced in time to improve litigation efficiency and reduce the burden of rights protection for investors.

The first line of defense for banks to resist risks is internal control. At present, internal control is mainly carried out by internal supervision, but it is far from enough. Banks should further consolidate and improve the platform construction through cooperation with audit institutions and other external institutions. Moreover, they should regularly check the perfection of the risk control system through the collaboration of the internal audit department and external audit institutions to ensure the safe and stable operation of the bank's credit assets [20].

#### 2.2.2. Review Risk Strategy

First of all, S Bank must review the borrower face to face and do an excellent job in the preloan inspection. The first hurdle of housing loan issuance is preloan inspection. Accurate and practical preloan assessment can effectively reduce the alarming debt rate and credit risk. This link determines whether the bank should lend to the borrower. If the bank lacks a perfect preloan inspection system and cannot accurately evaluate customers, it may lose some excellent customers. At the same time, it increases the housing credit risk [21]. At present, the main reason for the failure to repay the housing loan is that the borrower is unemployed. However, this phenomenon can be effectively avoided through the evaluation of the borrower. The person in charge of the bank's housing loan can understand the operation status of the borrower's enterprise through field investigation and evaluate the stability of the enterprise.

Second, the responsibility for postloan inspection should be apportioned to individuals. The postloan inspection of S Bank's housing loan is not standardized, and the inspection quality also needs to be improved. The person in charge of the postloan inspection of the bank even took the busy business as an excuse, did not track the postloan situation of the borrower in time, and only used static and straightforward text to describe the postloan inspection situation. This is a mere formality that cannot effectively analyze the borrower's repayment ability and capital flow. The borrower's self-reported economic capability cannot authoritatively prove their ability to repay the housing loan. Hence, S Bank should improve its postloan inspection system as soon as possible and assign responsibility to each related staff [22–24]. After issuing housing loans, S Bank should timely monitor the factors that may affect borrowers' repayment, comprehensively analyze the repayment possibility of borrowers, and form a written report to prevent credit risks effectively [25].

#### 2.2.3. Improving the Construction of Bank Risk Assessment System

Housing loan risk assessment is not only to manage the risks of a single borrower but also to optimize the allocation of risk capital and monitor and manage the overall risks faced by banks in combination with market policies and the situation of developers. Therefore, developing and establishing an internal evaluation model and evaluation system are essential [26].

The default loss rate and default probability of bank housing loans can be predicted in advance through statistical models. The models can accurately grasp borrowers' management, interest rate, and policy risks to reasonably forecast the possible dangers in the future [27]. Meanwhile, in establishing internal rating models and indicators, local policies and house prices should be taken into account. In addition, the evaluation system should be improved in combination with the borrower's historical credit information and personal data, which should be used as an essential basis for credit business development [28, 29].

#### 2.2.4. Addressing Interest Rate Risk

Interest rate risk will gradually appear with the promotion of market economic reform. S Bank should pay attention to the prevention of interest rate risk.

First, S Bank should adjust the interest rate of housing loans according to the fluctuation and adjustment cycle of interest rate, transfer the interest rate risk through interest rate adjustment, and improve the matching of the deposit term. Second, the credit risk of S Bank can be transmitted by increasing the interest rate pricing discount. S Bank shall first determine the loan interest rate discount of customers according to the qualifications of customers and developers and the cost of current market funds. When the market funds are relatively scarce, the bank can consider providing interest rate discounts for customers who need loans. When the borrower has credit problems, the bank can consider increasing interest rate discounts for such customers to reduce credit risk and improve bank income. Third, the financial market is developing toward diversification; correspondingly, S Bank can hedge through financial derivatives such as exchange options and interest rate futures to realize the effective control of housing credit risk [30–32].

Credit risk control has a significant impact on household consumption plans.

The data used here come from the detailed information of 1,027 resident families in Xi'an, Shaanxi Province. The household structure, capital, income, and essential characteristics of the household head of these families are learned through a questionnaire and a door-to-door interview.

### 2.3. Variable Selection and Data Description

#### 2.3.1. Variable Selection

Result variable: according to the consumption level, household consumption is divided into three consumption modes: enjoyment consumption, development consumption, and survival consumption. Survival consumption refers to the necessary primary consumption of each family, such as medical treatment, housing, and family food expenditure. Developmental consumption includes education, transportation, and communication expenditure. Enjoyment consumption refers to luxury goods and family clothing expenditure. Therefore, there are four main outcome variables in the present work: total household consumption, enjoyment consumption, developmental consumption, and survival consumption.

Processing variable: if the resident family does not participate in credit, it is 0; otherwise, it is 1.

Covariates: this study uses the propensity score matching (PSM) method to compare households without housing loans and households with housing loans to analyze the impact of housing credit on household consumption plans. The PSM is a statistical method to process data from observational studies. There are many data biases and confounding variables in observational studies due to various reasons. The PSM method can precisely reduce the influence of these biases and confounding variables to make a reasonable comparison between the experimental group and the control group. This method is commonly used in medicine, public health, economics, and other fields. We take, for example, the study of the impact of smoking on public health in the field of public health. Researchers often get data from observational studies rather than randomized controlled trials because the behavior and outcomes of smokers, and those of nonsmokers, are readily observable. However, if a randomized controlled experiment is to be conducted, it is not easy to enroll a large number of subjects and then randomly assign them to a smoking group and a nonsmoking group, and it is not in line with scientific research ethics. Observational research is the most appropriate research method in this case. However, unadjusted data from the most readily available observational studies can easily lead to erroneous conclusions. For example, it is concluded that smoking has no negative health effects by comparing some of the healthiest people in the smoking group with some of the poorest people in the nonsmoking group. The reason is analyzed from a statistical point of view. From a statistical point of view, this is because the observational study did not use randomization, and it is impossible to weaken the influence of confounding variables between the experimental group and the control group based on the effect of the law of large numbers, resulting in systematic bias. The PSM is used to solve this problem and remove the confounding factors between groups. In this study, the characteristics of the head of a family play a critical role in the risk appetite of the whole family. The credit funds may be used for investment consumption; the risk-neutral household head may obtain a certain interest by saving the credit funds. The total population of a resident household plays a decisive role in household consumption.

#### 2.3.2. Descriptive Statistics

The variables involved in this study and the statistical analysis results of variables are summarized in Table 1 and Figure 4.

According to Figure 4, in the sample statistical results, the average value of age is relatively high, while the average value of other factors is relatively low. In addition, the standard deviation of user age is also relatively large, around 8, while the standard deviation of other factors is around 1. Finally, the gap between the maximum and minimum user age is large, while the gap between other factors is small.

#### 2.3.3. Settings of the Measurement Model

The model reported here to estimate the impact of housing credit on household consumption level is described as follows:

(1) $$\begin{array}{c} \text{In}C_{ik}^{*}=a_{i}x_{i}+\eta w_{i}^{*}+\varepsilon . \end{array}$$

(2) $$\begin{array}{c} PC=E\left(C_{ik}^{1}-C_{ik}^{0}|w_{i}^{*}=1,X=x\right). \end{array}$$

(3) $$\begin{array}{c} NPC=E\left(C_{ik}^{1}-C_{ik}^{0}|w_{i}^{*}=0,X=x\right). \end{array}$$

(4) $$\begin{array}{c} TS=E\left(C_{ik}^{1}-C_{ik}^{0}X=x\right), \end{array}$$

where *C*_*ik*_^0^ and *C*_*ik*_^1^ represent the consumption of sample households not participating in and participating in housing credit, PC and NPC denote the average processing effect of sample households participating in and not participating in housing credit, and *TS* stands for the expected processing effect of randomly selecting a resident family sample from all resident family samples.

### 2.4. Correlation Test Analysis

#### 2.4.1. Ordinary Least Squares (OLS) Robustness Test of Household Consumption

Table 2 provides the OLS robustness test regression results of household consumption.

In Table 2, *∗∗* and *∗∗∗* indicate significant and very significant. The age of the head of household has a negative effect on all kinds of consumption in households, and the negative impact on the enjoyment consumption of households is significant at the level of 5%. This result shows that the age of the head of the household significantly affects the consumption of households. In the case of participating in housing credit, the health of the household head will positively affect the enjoyment consumption and developmental consumption within the family. The negative impact on the household survival consumption and total consumption is significant at the level of 1% and 10%, respectively. The educational level of the head of household will promote the enjoyment consumption and development consumption of the household, and its positive impact is significant at the level of 1%. From the perspective of family characteristics, the population size of households will promote the survival consumption and total consumption of households but will correspondingly reduce the developmental consumption of households. The positive impact on enjoyment consumption is significant at the level of 5%.

#### 2.4.2. Common Support Domain Condition

Whether the matching result is credible is mainly reflected by the standard support domain between the processing and control groups. A small coincidence area of the same covariates between the resident families participating in housing credit and those not participating in housing credit will effectively match the resident families participating in housing credit and those not participating in housing credit in the coincidence area of covariates. As a result, the matching accuracy is reduced.  Figure 5 illustrates the nuclear density of residents' family enjoyment, developmental, survival, and total consumption.

As shown in Figure 5, the matching degree adjustment for users is very effective under the consumption of PSM. Among them, the best matching adjustment effect is the enjoyment of consumer users, followed by the survival of consumer users, then the development of consumer users, and finally the total household consumption. The matching degree of various types of consumer users varies from the initial maximum difference of about 0.2 to the maximum difference of about 0.1 after the adjustment of the matching degree. It can be seen that the effect of the matching operation of the consumption propensity score is better.

#### 2.4.3. Balance Test

Based on the standard support test, the balance of the sample data is simultaneously tested. The balance test is conducted on residents' families participating or not participating in credit through three ways: nearest neighbor, radius, and kernel matching. The results are shown in Table 3 and Figure 6 below.

Within the effective range, the minimum value of mean deviation is 0, and the maximum value is 20%. The minimum value of B is 0, and the maximum value is 25%. The minimum value of *R* is 0.5, and the maximum value is 2. Combined with Table 2 and Figure 6, it can be seen that the enjoyment consumption, developmental consumption, survival consumption, and total household consumption are within the effective range, proving an excellent matching effect. Therefore, the balance test results show that the PSM method can effectively reduce the dominant deviation between the covariates of the control group and the treatment group, to effectively enhance the matching degree of sample data.

### 2.5. Analysis of PSM Matching Results

Since the regression results of the three methods of nearest neighbor, radius, and kernel matching are generally consistent, this study primarily describes the results of radius matching. This study uses the algorithm of equations (1)∼(2) to calculate and describe each factor.  Table 4 shows the specific results.

*PC*, *NPC*, and *TS* in Table 4 represent the average processing effects of resident families' participating credit, nonparticipating credit, and total samples, respectively. As shown in Table 4, the matching results of total household consumption under the three modes are *PC* < *NPC* < *TS*, and the radius matching results are 0.013, 0.052, and 0.125; the matching results of family enjoyment consumption under the three modes are *PC* < *NPC* < *TS*, and *PC* is significant at the 5% level under the nearest-neighbor matching, indicating that the negative impact of participation in credit on household enjoyment consumption is significant at the level of 5%. To a certain extent, the happiness of a family can be reflected by the enjoyment consumption of the family. Still, Table 4 demonstrates that the enjoyment consumption of resident families participating in credit is higher than that of resident families not participating in credit, indicating that the pressure brought by credit has a specific impact on the consumption of resident families. The matching results of family development consumption under the three modes are *PC* < *NPC* < *TS*. In addition, compared with the resident families who do not participate in credit, the developmental consumption of the resident families who participate in credit is improved to a certain extent. The value of *NPC* under the radius matching is significant at the 1% level. This indicates that the positive impact of nonparticipating credit on the resident families is significant at the 1% level. The matching results of family survival consumption under the three modes are *PC* < *NPC* < *TS*, demonstrating that the expected processing effect of the development consumption of the randomly selected family affected by credit is the largest. Meanwhile, the value of *NPC* under the radius matching is significant at the 1% level, indicating that the positive impact of nonparticipation in credit on resident families is significant at the 1% level.

### 2.6. Analysis of PSM of the Educational Level

Due to the differences in the life cycle of households, there are also certain differences in the consumption decisions of households in different periods, and the consumption thinking, consumption expectations, consumption concepts, and other factors of residents will have a certain impact on the consumption decisions of households. This study finds that the educational level of residents has the most obvious influence on their consumption decisions and has a guiding role in the consumption behavior of residents. The higher the education level of residents, the more mature their consumption concepts and psychology, and the higher the acceptance of new consumption models such as online consumption and credit. Therefore, this study takes the education level as the basis of investigation, examines the credit participation of residents, and calculates the content of the investigation according to the algorithm of equations (1) ∼ (4).  Table 5 presents the results.

According to Table 5, if the head of household is illiterate or semi-illiterate, the *PC* coefficient of total household consumption is -0.064, the *NPC* coefficient is 0.067, and the *TS* coefficient is 0.174; the *PC*, *NPC*, and *TS* coefficients of enjoyment consumption are -0.069, 0.163, and 0.405, respectively; the *PC*, *NPC*, and *TS* coefficients of developmental consumption are 0.046, 0.293, and 0.548, respectively; the *PC*, *NPC*, and *TS* coefficients of survival consumption are 0.058, 0.147, and 0.235, which all satisfy *PC* < *NPC* < *TS*. These results indicate that participating in credit will improve resident families' enjoyment, developmental, survival, and total consumption level.

When the educational level of the head of household is primary school or junior middle school, the *PC* coefficient of total household consumption is -0.026, the *NPC* coefficient is 0.017, and the *TS* coefficient is 0.105; the *PC*, *NPC*, and *TS* coefficients of enjoyment consumption are -0.136, -0.104, and -0.068, respectively; the *PC*, *NPC*, and *TS* coefficients of development consumption are 0.015, 0.085, and 0.217, respectively; the *PC*, *NPC*, and *TS* coefficients of survival consumption are -0.048, -0.018, and 0.058, respectively.

When the educational level of the head of household is high school or above, the *PC*, *NPC*, and *TS* coefficients of total household consumption are 0.084, 0.073, and 0.064; the *PC*, *NPC*, and *TS* coefficients of enjoyment consumption are 0.061, 0.053, and 0.048, respectively; the *PC*, *NPC*, and *TS* coefficients of development consumption are 0.147, 0.147, and 0.132 respectively; the *PC*, *NPC*, and *TS* coefficients of survival consumption are 0.095, 0.083, and 0.068, all in accordance with *PC* < *NPC* < *TS*.

## 3. Conclusions

The housing credit market highly concentrates capital and funds and is closely related to the development of the national economy. It is conducive to promoting economic development and optimizing the industrial structure. At the same time, the housing credit market has high risks. Especially in the current situation of serious information asymmetry and incomplete market development, the housing credit risk will have a great impact on the healthy development of the housing credit market. The development of blockchain technology provides new ideas for solving the problem of information asymmetry in bank credit management, thereby reducing bank operating costs and reducing credit risks. This study builds a bank housing credit blockchain alliance system to strengthen bank housing credit risk control based on the technical characteristics of blockchain. First, the application advantages of blockchain in the bank's housing credit business are analyzed according to its characteristics and system architecture. Then, the bank's housing credit risk control strategy is put forward on this basis. Finally, the mathematical model is used to explore the difference between the households that have obtained housing credit funds and the households that have not obtained housing credit funds in the expenditure of subsistence consumption and development consumption and enjoyment consumption. Under the adjustment of the PSM method, the enjoyment, development, survival, and total household consumption are all within the valid range and have a good matching effect. The results of the balance test demonstrate that the PSM method can effectively reduce the obvious deviation between the covariates of the control group and the treatment group, effectively enhancing the matching degree of the sample data. However, it is difficult for the blockchain system to balance the problems of high efficiency, high energy consumption, and database storage space due to the immature blockchain technology at present. These problems restrict the practical application of blockchain technology. Therefore, future research will further optimize blockchain technology to expand its application range.

## Figures and Tables

**Figure 1:** Blockchain data structure.

**Figure 2:** Overall functional architecture of the blockchain system.

**Figure 3:** Bank housing credit risk control strategy.

**Figure 4:** Variable statistical results ((a): mean; (b) standard deviation; and (c) maximum and minimum).

**Figure 5:** Kernel density function diagram (a): results of enjoying consumption before PSM; (b): results of enjoying consumption after PSM; (c): results of developmental consumption before PSM; (d): results of developmental consumption after PSM; (e): results of survival consumption before PSM; (f): results of survival consumption after PSM; (g): results of total household consumption before PSM; (h): results of total household consumption after PSM.

**Figure 6:** R-value of balance test (a): total household consumption; (b) enjoyment consumption; (c) developmental consumption; and (d) survival consumption.

**Table 1:** Variable description.

Variable serial number	Variable name	Variable description
(1)	Enjoyment consumption	Add 1 to the variable and take the logarithm
(2)	Developmental consumption	Add 1 to the variable and take the logarithm
(3)	Survival consumption	Add 1 to the variable and take the logarithm
(4)	Total household consumption	Add 1 to the variable and take the logarithm
(5)	Per capita consumption	Add 1 to the variable and take the logarithm
(6)	Age	Age of head of the household (years old)
(7)	Health level	If the householder is healthy, his health level is recorded as 1, and if he is not healthy, it is recorded as 0.
(8)	Degree of education	Education level of head of the household: illiterate = 0; primary school = 1; junior high school or above = 2
(9)	Family size	Total population within the family (people)
(10)	Labor force	Total number of the labor force within the family (people)
(11)	Number of students	Number of students in the family (people)
(12)	Number of elderly	Number of people who have lost their labor force within the family (people)
(13)	Total household income	Add 1 to the variable and take the logarithm
(14)	Participation in housing credit	Participation in housing credit is recorded as 1; if it does not participate in housing credit, it will be recorded as 0

**Table 2:** The OLS robustness test regression results of household consumption.

Variable	Enjoyment consumption	Developmental consumption	Survival consumption	Total household consumption
Age of head of the household	−0.005^∗∗^	−0.004	−0.002	−0.002
	(0.003)	(0.002)	(0.003)	(0.002)

Health level	0.085	0.067	−0.121^∗∗∗^	−0.054^∗^
	(0.064)	(0.072)	(0.039)	(0.037)

Degree of education	0.138^∗∗∗^	0.131^∗∗∗^	−0.029	0.016
	(0.036)	(0.041)	(0.027)	(0.028)

Family size	0.124^∗∗^	−0.037	0.041	0.038
	(0.055)	(0.051)	(0.037)	(0.031)

Labor force	0.002	0.086	0.072^∗^	0.064^∗∗^
	(0.065)	(0.061)	(0.037)	(0.034)

Number of students	−0.037	0.339^∗∗∗^	0.042	0.091^∗∗∗^
	(0.051)	(0.058)	(0.035)	(0.037)

Number of elderly	−0.047	−0.014	0.012	0.009
	(0.057)	(0.062)	(0.037)	(0.035)

**Table 3:** Balance test results.

Total household consumption				
Before matching		Nearest-neighbor matching	Radius matching	Kernel matching
Mean deviation	65.2	3.4	3.2	3.3
LR statistics	425.76	16.72	14.67	15.83
Pseudo-R2	0.315	0.012	0.006	0.012
B	142.6^*∗*^	23.8^*∗*^	23.1^*∗*^	23.3^*∗*^

*Enjoyment consumption*				
Mean deviation	66.7	3.2	4.1	3.5
LR statistics	425.87	11.65	15.97	12.59
Pseudo-R2	0.307	0.006	0.017	0.008
B	142.6^*∗*^	20.5^*∗*^	24.7^*∗*^	21.5^*∗*^

*Developmental consumption*				
Mean deviation	64.7	3.5	4.1	3.4
LR statistics	424.25	19.02	18.58	14.75
Pseudo-R2	0.306	0.011	0.011	0.008
B	141.4^*∗*^	24.9^*∗*^	24.8^*∗*^	22.5^*∗*^

*Survival consumption*				
Mean deviation	66.5	4.2	3.6	3.9
LR statistics	425.79	11.58	16.24	12.71
Pseudo-R2	0.312	0.006	0.010	0.007
B	141.7^*∗*^	20.1^*∗*^	24.1^*∗*^	21.2^*∗*^

**Table 4:** PSM matching results.

		*PC*	*NPC*	*TS*
Nearest-neighbor matching	Total household consumption	−0.054 (0.045)	−0.000 (0.025)	0.097^*∗∗*^ (0.045)
	Enjoyment consumption	−0.107^*∗∗*^ (0.052)	−0.045 (0.051)	0.084^*∗*^ (0.050)
	Developmental consumption	−0.064 (0.062)	0.058 (0.092)
	Survival consumption	−0.007 (0.042)	0.024 (0.032)	0.071 (0.081)

Radius matching	Total household consumption	0.013 (0.026)	0.052^*∗∗*^ (0.022)	0.125^*∗∗∗*^ (0.031)
	Enjoyment consumption	−0.032 (0.051)	0.019 (0.050)	0.105 (0.057)
	Developmental consumption	0.075^*∗*^ (0.046)	0.164^*∗∗∗*^ (0.042)	0.324^*∗∗∗*^ (0.067)
	Survival consumption	0.022 (0.027)	0.051^*∗∗*^ (0.021)	0.112^*∗∗∗*^ (0.027)

Kernel matching	Total household consumption	−0.018 (0.025)	0.026 (0.017)	0.114^*∗∗∗*^ (0.032)
	Enjoyment consumption	−0.066 (0.047)	−0.065 (0.046)	0.104 (0.067)
	Developmental consumption	0.028 (0.045)	0.029 (0.047)	0.295^*∗∗∗*^ (0.070)
	Survival consumption	−0.004 (0.025)	−0.004 (0.025)	0.097^*∗∗∗*^ (0.034)

**Table 5:** Matching results of propensity score of educational level group.

		*PC*	*NPC*	*TS*
Illiterate or semi-illiterate	Total household consumption	−0.064 (0.065)	0.067 (0.053)	0.174*∗∗* (0.076)
	Enjoyment consumption	−0.069 (0.147)	0.163 (0.127)	0.405*∗∗∗* (0.147)
	Developmental consumption	0.046 (0.159)	0.293*∗∗* (0.146)	0.548*∗∗∗* (0.163)
	Survival consumption	0.058 (0.053)	0.147*∗∗∗* (0.051)	0.235*∗∗∗* (0.074)

Primary or junior high school	Total household consumption	−0.026 (0.043)	0.017 (0.034)	0.105*∗∗∗* (0.036)
	Enjoyment consumption	−0.136*∗* (0.061)	−0.104 (0.074)	-0.068 (0.092)
	Developmental consumption	0.015 (0.063)	0.085 (0.050)	0.217*∗∗∗* (0.062)
	Survival consumption	−0.048 (0.036)	−0.018 (0.027)	0.058 (0.031)

High school and above	Total household consumption	0.084*∗* (0.049)	0.073*∗∗* (0.035)	0.064*∗* (0.032)
	Enjoyment consumption	0.061 (0.086)	0.053 (0.075)	0.048 (0.071)
	Developmental consumption	0.147 (0.094)	0.147*∗* (0.081)	0.132*∗* (0.074)
	Survival consumption	0.095*∗* (0.057)	0.083*∗∗* (0.047)	0.068*∗* (0.039)

## Data Availability

All data are fully available without restriction
